The article "Tuberculosis of the Lower Lumbar Spine with an Atypical Radiological Presentation - A Case Mimicking a Malignancy -" was published in 2007. Journal: Asian Spine J.

# Tuberculosis of the Lower Lumbar Spine with an Atypical Radiological Presentation - A Case Mimicking a Malignancy -

**DOI:** 10.4184/asj.2007.1.2.102

**Published:** 2007-12-31

**Authors:** Juhae Jahng, Young-Hoon Kim, Kyo-Sun Lee

**Affiliations:** Department of Orthopedic Surgery, Catholic Medical College, The Catholic University of Korea, Seoul, Korea.

**Keywords:** Atypical tuberculosis, Spondylitis, Malignancy

## Abstract

A 65-year-old woman was treated for an atypical radiological presentation of spinal tuberculosis. Compared with previously reported cases, the following two different radiographic features were found. 1) Although there was multiple and skipped involvement of the vertebral body, the intervertebral disc was relatively preserved. 2) The presence of an epidural granuloma indicated an epidural extension of the lesion of the adjacent vertebral body. These findings strongly mimicked bone marrow infiltrative disease such as a malignancy. Tuberculosis was confirmed through an open biopsy and the patient was treated successfully with antitubercular chemotherapy. This case highlights the importance of being aware that spinal tuberculosis has many different radiographic features and can mimic a spinal malignancy.

## Introduction

With the development of appropriate chemotherapy and advanced imaging techniques, most cases of spinal tuberculosis are readily diagnosed and are treated successfully. However, as previously reported, an atypical radiological presentation of spinal tuberculosis presents a challenge for an appropriate diagnosis and early treatment, due to the atypical clinical and radiographic features^1^,^2^. Several different features of atypical radiological presentation of tuberculosis have been described and reported^1^,^3^-^6^. We encountered a unique case of clinical and radiographic atypical spinal tuberculosis that mimicked the findings of a spinal malignancy.

## Case Report

A 65-year-old woman presented with a three-month history of aggravating low back and leg pain. At the first examination, the patient had tenderness over the lower lumbar and tension signs on the lower lumbar nerve. There was hypesthesia on the lateral aspect of both lower legs with no definite motor deficits. Laboratory studies showed a high erythrocyte sedimentation rate of 110 mm/hr (normal 0-15 mm/hr), C-reactive protein level of 9.3 mg/dL (normal 0-0.5 mg/dL) and a mild increase in the levels of liver enzymes and level of normal alkaline phosphatase. Tumor markers checked initially were normal. A plain film of the chest demonstrated evidence of prior-healed tuberculosis. A plain radiograph of the lower lumbar spine showed spondylotic changes without a destructive lesion of the vertebral column (Fig. 1). Advanced radiographic studies were performed with a first impression of spinal stenosis or other infectious condition of the spinal column. Magnetic resonance imaging (MRI) revealed several infiltrative lesions with low signal intensity on the T1 weighted images, and isointensity on a T2 weighted image, mainly at L5 as well as at S1 and L1. The lesions were homogenously enhanced. In addition, at the L4-5 level, severe thecal sac and nerve root compression was observed resulting from the epidural mass anteriorly, hypertrophied ligament and facet posteriorly. However, the discs were relatively preserved (Fig. 2). Computerized tomography (CT) was performed. CT scans of these affected sites revealed a severe spinal stenotic condition without any definite destruction of the vertebral body (Fig. 3). From these clinical and radiological findings, a bone marrow infiltrative neoplasm was suspected; in particular, multiple myeloma or a metastasis. Decompression and a biopsy were performed with the aim of making a final diagnosis as well as palliation of the clinical symptoms. The surgical findings revealed the stenotic conditions to coincide with the preoperative radiographic findings. There was a friable soft epidural mass beneath the posterior longitudinal ligament. However, there was no evidence of infection or an abscess. A culture and biopsy for bacterial and tuberculosis were performed. A histological examination of the epidural mass and vertebral body from L5 showed an epitheloid granuloma with areas of central necrosis and the presence of Langhans giant cells (Fig. 4). A culture of the specimen revealed the presence of *Mycobacterium tuberculosis*. The patient was treated successfully with postoperative chemotherapy consisting of isoniazid, rifampicin, ethambutol and pyrazinamide.

## Discussion

Advances in diagnostic imaging and chemotherapy have led to successful treatment of spinal tuberculosis. Typical spinal tuberculosis, which has specific radiological findings of involvement of adjacent vertebral bodies with destruction of the intervening disc and a paravertebral soft tissue involvement, can be diagnosed easily and treated successfully^7^,^8^. However, spinal tuberculosis with atypical clinical and radiographic findings can result in a delayed diagnosis. The incidence of atypical spinal tuberculosis has been reported to be 2.1% in a recent study^2^. A variety of radiological features of atypical spinal tuberculosis can lead to a misdiagnosis and incorrect treatment, and in certain cases, can increase the risk of other complications such as a neurological deficit^9^,^10^.

Atypical features that were described in the previous reports are 1) involvement of the spinal posterior element with a sparing of the anterior column; 2) skip lesions; and 3) neural component compression as a result of tuberculosis granuloma^4^. The most common site of involvement of the posterior element of the spine is the pedicle^1^. Hematogenous spread of tuberculosis is thought to the primary event for pathogenesis. These posterior lesions would be distinguished from the metastatic lesions. The reason why the noncontiguous vertebrae were involved is unclear, but the unique venous system of the vertebra, as described by Batson^11^, is believed to be partly responsible. An intraspinal tubercular granuloma can present as an extradural or intradural tuberculoma with or without a bony abnormality^7^. An intraspinal, extradural tubercular granuloma is one of the atypical radiographic features of spinal tuberculosis that mimic a malignancy^5^,^6^,^12^. In our case, the involved lesions were multiple and skipped, which lead to spinal cord compression as a result of an epidural mass and co-existing spondylosis. Especially, even though involvement of the L5 vertebral body was advanced and L1, L5 and S1 were involved (not the thoracolumbar region), the intervertebral disc between L5-S1 was relatively preserved. Findings that involved a homogenously enhanced epidural mass with multiple signal changes in the bone marrow, preservation of the adjacent intervertebral disc, and no paraspinal abscess would result in a misdiagnosis of a malignancy or metastatic lesions.

This case shows that it is important to be aware that spinal tuberculosis has many different radiographic features and can mimic a spinal malignancy.

## Figures and Tables

**Fig. 1:** An anteroposterior and lateral radiograph of the lumbar spine shows the multilevel spondylosis with mild osteopenia of L5 body.

**Fig. 2:** (**A**) A sagittal T1-weighted magnetic resonance imaging scan shows low signal bone marrow infiltrations involving L1, 5 and S1 vertebral bodies. (**B**) On enhances imaging, the lesions were homogenously enhanced. (**C**) A sagittal T2-weighted scan shows isosignal intensity at the same lesion and preservation of intervertebral disc. There was no evidence of paravertebral abscess. (**D**) Axial scan shows the stenotic condition resulting from epidural mass and facet arthritis. There was no evidence of paravertebral soft tissue abnormalities.

**Fig. 3:** CT scan shows thecal sac compression without the destruction of bone or paravertebral absecess.

**Fig. 4:** This photomicrograph shows typical chronic granulomatous infection. (tissue from epidural mass) consisting of an epitheloid granuloma, caseous necrosis and Langhans' giant cell. (Hematoxylin-Eosin stain, A; ×100, B; ×400)
